# Analysis of the Effect of Incentive Nursing Intervention in Children with Severe Viral Encephalitis and Myocarditis during Rehabilitation Based on Diffusion Weighted MRI

**DOI:** 10.1155/2021/9993264

**Published:** 2021-05-13

**Authors:** Qiuai Ren, Li Guo, XiuLan Liu, PengFei Xiao, Shuifang Tang, Ashutosh Sharma, Tarandeep Singh Walia, Mohd Asif Shah

**Affiliations:** ^1^Weinan Vocational and Technical College, Weinan, China; ^2^Department of Educational Administration, Brain Hospital of Hunan, ChangSha 410007, China; ^3^Department of Emergency Medicine, Brain Hospital of Hunan, ChangSha 410007, China; ^4^Brain Hospital of Hunan, ChangSha 410007, China; ^5^Institute of Computer Technology and Information Security, Southern Federal University, Rostov-on-Don, Russia; ^6^School of Computer Application, Lovely Professional University, Phagwara, India; ^7^Bakhtar University, Kabul, Afghanistan

## Abstract

**Background:**

Severe viral encephalitis in children causes a viral infection that damages their central nervous system. This situation arises the mental abnormalities, sudden rise in body temperature, disturbance of consciousness, and so forth in children, which can be life-threatening.

**Objective:**

This work aimed at exploring the effect of diffusion weighted MRI on children with severe viral encephalitis and myocarditis.

**Methods:**

This work presents a diffusion weighted MRI scanning method that involves scanning through a serial imaging device, axial scanning, and sagittal and coronal scanning. 60 children with severe viral encephalitis and myocarditis who admitted to Brain Hospital of Hunan Province from April 2017 to May 2020 were deemed as research subjects. All the children underwent CT and MRI examination, blood routine examination, and cerebrospinal fluid examination after admission. This work uses the random number table method to classify the subjects into control group and observation group, each consisting of 30 cases. Children in the control group were provided with the routine nursing intervention, whereas children in the observation group were subjected to incentive nursing intervention. The baseline data, ECG monitoring indicators, body abnormalities, and clinical symptom relief time of the two groups of children were compared and the results of diffusion weighted MRI scans were analyzed and the ADC values were counted.

**Results:**

The two groups of children were compared on the basis of baseline data, and the variation was not statistically substantial (*P* > 0.05). The cases of children in the control group had higher heart rate and respiration, and physical dysfunction, language dysfunction, unconsciousness, and nervous dysfunction were more than those in the observation group. However, the cases of blood oxygen saturation were less than those of the observation group. After nursing intervention done for the control group, remission time of clinical symptoms such as convulsion, physical dysfunction, unconsciousness, and nerve dysfunction was longer relative to the observation group (all *P* < 0.05 are considered).

**Conclusion:**

The diffusion weighted MRI had diagnostic significance for severe viral encephalitis and myocarditis. For children with severe viral encephalitis and myocarditis, clinical incentive nursing intervention was particularly imperative. It can not only help children to relieve symptoms and control the deterioration of the disease in a short time but also help improve the quality of life of the children and the confidence of family members to cope with the disease.

## 1. Introduction

Viral encephalitis refers to brain inflammation caused by a virus directly invading the brain parenchyma. The main cause of this disease is enterovirus infection, which mainly includes polio virus, Coxsackie virus A and B, and Echo virus. The disease has the characteristics of seasonality, epidemic, and so forth. It mostly occurs in winter and spring and is often self-limiting [1]. Children's viral encephalitis mainly refers to the viral infection invading the pia mater and causing damage to the central nervous system. Children manifested with obvious mental abnormalities, sudden rise in body temperature, disturbance of consciousness, and so forth, which can be severely life-threatening. In the clinic, children with viral encephalitis are mostly classified into two types: mild type and critical type. Critically ill children are often complicated with myocarditis, which is clinically manifested as damage to brain and heart function at the same time [2]. Myocarditis refers to a disease in which localized or diffuse inflammatory lesions of the myocardium are the main manifestations, and the pathogenesis is not yet completely diagnosed. According to the investigation of rat samples, viral myocarditis can be divided into 3 stages. The virus invades myocardial cells to multiply through specific receptors, leading to myocardial necrosis. The continuous response can cause myocardial remodeling and eventually cause progressive heart failure. Most children are with severe arrhythmia, heart failure, and other clinical manifestations [3]. If the clinical treatment is not timely or the care is improper, it can lead to aggravated damage to the brain tissue or heart function of the child and have a serious impact on the growth and development of the child and the quality of life [4]. A basic block diagram of the entire research process for effective analysis of incentive nursing innovation based on diffusion weighted MRI is depicted in Figure 1.

In the developing countries, the literature survey suggests that approximately 50% to 60% patients are identified with the viral encephalitis and possess long-term prognosis [5–7]. This situation leads to a tremendous stress and financial burden on the families of patients and also on the society [8–12]. Thus, this scenario leads to the research for identification of prognosis factors in the patients suffering from viral encephalitis. The research is oriented towards the early decision-making and timely treatment for improving the capabilities of the framework in favor of patients while improving the living standard. This type of improvement in the research domain leads to the improved clinical diagnosis as well as social consequences. The epidemiological data should be considered for diagnosis along with the clinical indicators, previous medical history of the patients, and a comprehensive analysis of auxiliary examinations performed. The detection of brain tissues acts as a gold standard for the diagnosis of viral antigens or for determining the antibodies in cerebrospinal fluid. However, it should be noted that the diagnostic frequency of viral encephalitis is low around the world and still there are several cases that remain unknown [13–15].

Salazar et al. [16] presented a case study in which anti-N-methyl-D-aspartate receptor encephalitis is seen, which is related to the involuntary movement as well as hypersalivation symptoms. These situations can only be controlled by narcotics and other high-dosage sedation which is not at all good for patients' health. The authors suggested that the change in hypothalamic neurotransmitter levels can stimulate the parasympathetic neurons of nervous system. Taguchi et al. [17] presented an instance of viral encephalitis who already had a medical history of ovarian teratoma, which can be reduced using anesthetic drugs. It was found that patients having fever symptoms is very consistent in the literature [18–20] and the incidents of teratomas were also found to be common in the previous reports [21]. Comparative to the patients suffering from tumors, the consistency was found in the reoccurrence rates of the patients [22, 23]. The authors in [24] reported that the patients with MRI abnormalities have disorders like epilepsy, involuntary movement of the limbs, and other mental disorders, which can indicate the MRI related clinical severities. Therefore, they presented a specific mechanism for viral encephalitis as a further research challenge.

The review of literature for viral encephalitis reveals that the early diagnosis is of great significance for the clinical treatment and prognosis of children with viral meningitis and myocarditis. MRI is currently widely adopted in clinics due to its high tissue resolution. However, its sequence is simple, including only T1W1, T2W1, T2FLAIR, and enhanced scanning [25]. The new technology diffusion weighted MRI imaging is based on the movement of water molecules, which provides information based on the physiological state of the brain. The sensitivity of clinical diagnosis of acute cerebral infarction is as high as 94%, and the specificity is 100%. Moreover, it is also employed to distinguish between arachnoid cyst and epidermoid cyst, subdural empyema and effusion, abscess, and tumor necrosis. It can provide valuable information in the diagnosis and differential diagnosis of other intracranial lesions such as tumors, infections, trauma, and demyelination [26].

The objective of this work is to explore the diffusion effect in weighted MRI for children having symptoms of viral encephalitis and myocarditis. The major contributions of this article are heighted as follows:

- The diffusion weighted MRI scanning method is employed using a single-shot SE-EPI serial imaging device for scanning. A 9-channel head coil is adopted with layer thickness of 6 mm, spacing of 2 mm, and NEX = 3. The enhanced scan Meglumine acid was used for contrast agent gadolinium injection followed by axial, sagittal, and coronal scanning.
- The experimentation was conducted on 60 children with severe viral encephalitis and myocarditis symptoms between April 2017 and May 2020 who admitted to Brain Hospital of Hunan Province. The children underwent CT and MRI examination, blood routine examination, and cerebrospinal fluid examination, on the basis of which they were classified into control and observation groups, each with 30 cases. The children in the control group were provided with the routine nursing intervention, while children in the observation group were subjected to incentive nursing intervention.
- The baseline data, ECG monitoring indicators, body abnormalities, and clinical symptom relief time of the two groups of children were compared, and the appropriate nursing methods were selected according to the inspection results. The results of diffusion weighted MRI scans were analyzed and the ADC values were also computed, on the basis of which the diagnostic significance of diffusion weighted MRI for severe viral encephalitis and myocarditis is observed.
- This significant contribution can control the deterioration of the disease in a short time, thereby improving the living standard of the children and the confidence of family members to cope with the disease.

The rest of this article is organized as follows: research methods including the description of the subjects, research routes, and MRI analysis methods are discussed in Section 2.  Section 3 presents the research results trailed by the experimental discussion in Section 4.  Section 5 presents the concluding remarks along with future research directions.

## 2. Research Methods

This section provides a research route, research subjects along with diffusion weighted MRI scanning method and image analysis, nursing methods, observation indicators, and the information of statistical software.

### 2.1. Research Route

For the effective analysis of incentive nursing innovation based on diffusion weighted MRI, the research route for this work is described in Figure 2.

This research route is designed to analyze the effect of incentive nursing innovation based on diffusion weighted MRI in the children suffering from viral encephalitis and myocarditis. The method is initially applied on sixty children with the symptoms of viral encephalitis and myocarditis, and MRI diffusion is performed. Based on the result analysis of diffusion process, the control group and the observation group are formed. The control group is provided with the routine nursing intervention and the observation group is subjected to the incentive nursing intervention. The results of both groups are compared and the effect of MRI intervention is analyzed and summarized.

### 2.2. Research Subjects

A total of 60 children with severe viral encephalitis and myocarditis were selected from Brain Hospital of Hunan Province from April 2017 to May 2020. All the children underwent CT and MRI examination, blood routine examination, and cerebrospinal fluid examination after admission. This work uses the random number table method to classify the subjects into control group and observation group, each consisting of 30 cases. The control group comprises 21 male children and 9 female children. The age ranged from 4 months to 8 years, with an average of 3.09 ± 1.42 years of age. However, the observation group comprises 20 male children and 10 female children. The age was 3 months to 9 years, with an average of 3.16 ± 1.39 years of age. The general data is not statistically significant based on the gender and age of both groups and, therefore, they are comparable. The medical ethics committee of Brain Hospital of Hunan Province studied and approved this investigation. The relevant diagnostic criteria of severe viral encephalitis in “*Diagnosis and Treatment of Children's Viral Encephalitis*” and the related content of myocarditis in “*Diagnostic Criteria of Viral Myocarditis*” were discussed. The inclusion criteria are as follows: the patients who met the above-mentioned conditions and have not received any other treatment in the recent years; and family members of the children knew and signed the informed consents. The exclusion criteria are as follows: the patients who suffer from any sort of immune system diseases, those with other nonviral infections in the cranium, those who were allergic to the relevant treatments used in this investigation, and those with poor compliance to this investigation.

### 2.3. Diffusion Weighted MRI Scanning Method and Image Analysis

The scanning was conducted by a single-shot SE-EPI sequence imaging device, and a 9-channel head coil was employed, which mainly included inversion recovery sequence, fast spin echo, and water suppression sequence, with layer thickness of 6 mm, spacing of 2 mm, and NEX = 3. During the enhanced scan, the child needed to be injected with the contrast agent gadopentetate meglumine injection at a dose of 0.1 mmol/kg. After injection, scan was performed in axial, sagittal, and coronal positions. If the child cannot cooperate, he/she needed to drink 5% water and 1 mL/kg of chloric acid half an hour before the scan.

When the scan results were analyzed, two experienced diagnostic physicians evaluated them separately. If the evaluation results of the two were inconsistent, a third, more senior imaging physician would conduct the diagnostic evaluation. The specific content included the location, number, size, and scope of the lesion. ADC measurement was implemented via the ADC statistical software, the lesion and the normal brain tissue on the opposite side were measured, and finally the average result was calculated.

### 2.4. Nursing Methods

According to the results of diffusion weighted MRI scans, children in the control group are provided with the routine nursing intervention. It mainly included the monitoring of the vital signs, consciousness state, and physical activity of the child. The child's family members were informed of the disease-related knowledge and the current treatment of the child. Incentive nursing intervention was given to children in the observation group. The content of routine nursing was the same as that of the control group, and psychological nursing and rehabilitation nursing were also implemented. In daily nursing, nurses should communicate with children and their families more, be familiar with the children's hobbies, establish a friendly care relationship with the children, and use touch, whisper, and other methods to comfort the children. In addition, it was necessary to comfort and encourage the children's family members and promptly inform them with the treatment results. Parents should understand the necessity of treatment, maintain an optimistic attitude, actively respond, and cooperate with the doctor to help the children recover as soon as possible. Rehabilitation care was performed to help children perform more physical activities, including upper and lower limb exercises, wrists, elbows, fingers, hips, knees, and ankle joints, 3 times a day.

### 2.5. Indicators for the Observation

- The baseline data of the control and the observation groups of the children were compared.
- Diffusion weighted MRI scan results of severe viral encephalitis and myocarditis were analyzed, and the ADC value was calculated.
- The ECG monitoring indicators of the two groups of children were compared, including heart rate, respiration, and blood oxygen saturation.
- The number of cases of physical abnormalities in the two groups of children were compared, including physical impairment, language impairment, and intellectual impairment.
- The clinical symptoms relief times of the two groups of children after the incentive nursing intervention were compared, including convulsions, physical dysfunction, unconsciousness, and nerve dysfunction.

### 2.6. Statistical Software

The data analysis in this work is done employing the SPSS 22.0 statistical software. The percentage count of the data is considered and the chi-square test is done for the comparison between these groups. The statistical significance of the data is inferred using the *P* value (*P* < 0.05). It tests the variance between the data groups which are to be measured at the ordinal or continuous level. This test does not need the data to be normally distributed and can be applied to a group of random samples from the entire population. The chi-square test statistics rank the data using the chi-square distribution for computing the significant *P* values. This test is useful in controlling the experimental variability of data and can be applied to the group of random samples without checking the normality distribution of the dataset being used. The *P* values of the test should be significantly less than 0.05 as the smaller *P* value of this test is suggestive of selection of the entire data for the analysis. The comparative analysis is done to demonstrate the feasibility of the presented method utilizing the nonparametric data statistics.

## 3. Results

The experimental analysis of diffusion weighted MRI scanning method and image analysis for discussing the effects of incentive nursing intervention in children with severe viral encephalitis and myocarditis during rehabilitation are provided in this section.

### 3.1. Comparative Analysis of Baseline Data

The control group contains the patients who are given the nursing intervention and the observation group contains the patients who are provided with the incentive nursing intervention. Both groups are compared on the basis of data.  Figure 3 shows that the baseline data of both groups were compared, and the statistical implication of the difference was found to be not significant enough as *P* > 0.05.

This comparison reveals that the baseline data contain both male and female children of varying age groups. The numerical value of male children is higher than that of the female children, and they are evenly distributed into control and observation groups.

### 3.2. Diffusion Weighted MRI Scan Results

Diffusion weighted MRI scans showed that the brain lesions of the children mostly involved the subcortex, thalamus, and midbrain. Figures 4 and 5 illustrate that the lesions were patches or large patches with slightly longer T1, while the lesions in the brain and heart areas showed obvious hyperintensity.

The results of diffusion weighted MRI scans were analyzed in terms of ADC values to determine the diagnostic significance of diffusion weighted MRI for severe viral encephalitis and myocarditis. The ADC value of the severely infected portion was considerably lower as compared to the healthier part as shown in Figure 6. The statistical implication of the difference is significant enough as the significant value comes out to be *P* < 0.05.

### 3.3. Comparison of ECG Monitoring Indicators between Two Groups of Children

After comparison, the heart rate and respiration of children in the control group were significantly higher than those of the observation group (Figure 7), while the blood oxygen saturation was lower for this group. The difference was substantial in terms of this statistical significance (*P* < 0.05).

### 3.4. Comparison of the Number of Abnormalities in the Two Groups of Children

After comparison, the number of cases in the control group having physical, language, and intellectual dysfunctions was more than that in the observation group (Figure 8), and the variation has statistical significance (*P* < 0.05).

### 3.5. Comparison of Clinical Symptom Remission Time

After nursing intervention, in the control group, the remission time of clinical symptoms such as convulsion, physical dysfunction, unconsciousness, and nerve dysfunction was longer compared to that in the observation group, and the variation was remarkable statistically providing the significance value of *P* < 0.05, as illustrated in Figure 9.

## 4. Discussion

Severe viral encephalitis is a fatal intracranial infectious disease, in which the virus directly destroys the brain parenchyma and induces neuropathy. Imaging examination reveals diffuse or focal changes in neuronal deformation and necrosis, as well as severe damage to functional areas. Normal cell metabolism in the brain is disordered, and a large amount of necrosis occurs [27]. Some children may have cerebral edema myocarditis. The cardiac function of children with myocarditis is obviously seriously affected, causing the children to have obvious physical fatigue, palpitations, and other discomforts. Severe children may also have heart failure, shock, and so forth, and some children may even die suddenly. Therefore, in clinical nursing work, the observation of the patient's condition is the top priority [28].

The nursing work was carried out based on the results of diffusion weighted MRI. Diffusion weighted MRI imaging reflects tissue information by measuring the motion of water molecules in vivo. It can clearly distinguish cytotoxic edema from vasogenic edema, so it has significant advantages and has been clinically applied in the diagnosis of intracerebral diseases [29]. In this work, diffusion weighted MRI scan revealed that brain lesions mainly involved subcortex, thalamus, and midbrain, and the lesions were patches or large patches slightly longer than T1. The lesions in brain and heart showed high signal intensity. With severe viral encephalitis as an example, as the disease progresses, the scope of cerebral vasogenic edema gradually expands. At this time, cytotoxic edema in the lesion still exists, and the two coexist. When scanned by diffusion weighted MRI, vasogenic edema produces transmission effect, while ADC value can remove this effect and reduce imaging error, so it has practical value.

At present, the domestic treatment of severe viral encephalitis and myocarditis has achieved remarkable results. Most of the children can recover as long as they receive timely clinical treatment, but there are still some children who have various adverse reactions, even disability and death, which increase the burden on the children and their families. Studies suggested that effective nursing intervention was of great significance for the recovery of children after treatment [30–32]. Therefore, according to the results of imaging examination, two different nursing modes were implemented for the children to compare their effects. The outcomes obtained for heart rate and respiration of the children in the control group are higher than those in the observation group, while the saturation of oxygen is lower than that in the observation group. Additionally, the physical, language, and mental dysfunctions in the children of the control group were higher than those in the observation group. After clinical nursing intervention, the time of remission for clinical symptoms, convulsion, physical dysfunction, unconsciousness, and nerve dysfunction, in the control group was greater than that in the observation group.

## 5. Conclusion

This work contributed to the analysis of diffusion effect in weighted MRI for children having symptoms of viral encephalitis and myocarditis. The experimentation was conducted on 60 children who admitted to Brain Hospital of Hunan Province with the symptoms of viral encephalitis or myocarditis. These children underwent the CT and MRI examination and are divided into control and observation groups for analysis. The various experimental analyses were performed on the baseline data using the ECG monitoring indicators and body abnormalities, and clinical symptom relief times of the two groups of children were compared. Using the nursing intervention, the remission times of clinical symptoms such as convulsion, physical dysfunction, unconsciousness, and nerve dysfunction were observed to be statistically significant having *P* < 0.05.

In summary, diffusion weighted MRI had great significance for the diagnosis of severe viral encephalitis and myocarditis. For children with severe viral encephalitis and myocarditis, clinical incentive nursing intervention was particularly imperative, which helped children relieve symptoms in a short period of time and control the deterioration of their condition. Moreover, it also helped to improve the living standard of children and the confidence of family members in coping with the disease, which was worthy of further clinical promotion and adoption. This investigation uses the smaller sample size, which certainly affects the research results; therefore, the future perspective of this work requires the expansion of sample size for the establishment of incentive nursing intervention-based algorithms in the current scenario.

## Figures and Tables

**Figure 1:** Block diagram for effective analysis of incentive nursing innovation.

**Figure 2:** Research route.

**Figure 3:** Comparative analysis of the baseline data.

**Figure 4:** Severe viral encephalitis.

**Figure 5:** Myocarditis.

**Figure 6:** ADC value.

**Figure 7:** ECG monitoring indicators.

**Figure 8:** Number of cases of body abnormalities.

**Figure 9:** Remission time of clinical symptoms.

## Data Availability

All data are shared in the main manuscript.

## References

[1] Adenot M., Frobert E., Blanchard G. (2014). Clinical presentation of severe viral encephalitis with known causative agents in children. *Journal of Child Neurology*.

[2] Inui Y., Yakushijin K., Okamura A., Tanaka Y., Shinzato I. (2019). Human herpesvirus 6 encephalitis in patients administered mycophenolate mofetil as prophylaxis for graft‐versus‐host disease after allogeneic hematopoietic stem cell transplantation. *Transplant Infectious Disease*.

[3] Koeller K. K., Shih R. Y. (2017). Viral and prion infections of the central nervous system: radiologic-pathologic correlation:from the radiologic pathology archives. *Radiographics*.

[4] Chen Y. F., Hu L., Xu F., Liu C. J., Li J. (2019). A case report of a teenager with severe hand, foot, and mouth disease with brainstem encephalitis caused by enterovirus 71. *BMC Pediatrics*.

[5] Raschilas F., Wolff M., Delatour F. (2002). Outcome of and prognostic factors for herpes simplex encephalitis in adult patients: results of a multicenter study. *Clinical Infectious Diseases*.

[6] Dhiman G., Oliva D., Kaur A. (2021). BEPO: a novel binary emperor penguin optimizer for automatic feature selection. *Knowledge-Based Systems*.

[7] Erlanger T. E., Weiss S., Keiser J., Utzinger J., Wiedenmayer K. (2009). Past, present, and future of Japanese encephalitis. *Emerging Infectious Diseases*.

[8] Solomon T. (2006). Control of Japanese encephalitis - within our grasp?. *New England Journal of Medicine*.

[9] Dhiman G., Singh K. K., Soni M. (2021). MOSOA: a new multi-objective seagull optimization algorithm. *Expert Systems with Applications*.

[10] Venkatesan A. (2015). Epidemiology and outcomes of acute encephalitis. *Current Opinion in Neurology*.

[11] Poongodi M., Sharma A., Vijayakumar V. (2020). Prediction of the price of Ethereum blockchain cryptocurrency in an industrial finance system. *Computers & Electrical Engineering*.

[12] Rathee G., Sharma A., Kumar R., Ahmad F., Iqbal R. (2020). A trust management scheme to secure mobile information centric networks. *Computer Communications*.

[13] Lohitharajah J., Malavige N., Wanigasinghe J., Gamage R., Gunaratne P. ., ..., Chang T. (2017). Viral aetiologies of acute encephalitis in a hospital-based South Asian population. *BMC Infectious Diseases*.

[14] Srihari K., Dhiman G., Somasundaram K., Sharma A., Rajeskannan S. ., ..., Masud M. (2021). Nature-inspired-based approach for automated cyberbullying classification on multimedia social networking. *Mathematical Problems in Engineering*.

[15] Feng G., Zhou L., Li F., Hu Y., Wang X., Tian X. (2020). Predictors of outcome in clinically diagnosed viral encephalitis patients: a 5-year prospective study. *BioMed Research International*.

[16] Salazar R., James E., Elsayed M. (2012). Profuse sialorrhea in a case of anti N-methyl-D-aspartate receptor (NMDAR) encephalitis. *Clinical Neurology and Neurosurgery*.

[17] Taguchi Y., Takashima S., Nukui T., Tanaka K. (2010). Hypersalivation in a patient with anti-NMDAR encephalitis with ovarian teratoma. *Internal Medicine*.

[18] Miya K., Takahashi Y., Mori H. (2014). Anti-NMDAR autoimmune encephalitis. *Brain and Development*.

[19] Peery H. E., Day G. S., Dunn S. (2012). Anti-NMDA receptor encephalitis. The disorder, the diagnosis and the immunobiology. *Autoimmunity Reviews*.

[20] Gabilondo I., Saiz A., Galán L. (2011). Analysis of relapses in anti-NMDAR encephalitis. *Neurology*.

[21] Wang R. J., Chen B. D., Qi D. (2015). Anti-N-methyl-D-aspartate receptor encephalitis concomitant with multifocal subcortical white matter lesions on magnetic resonance imaging: a case report and review of the literature. *BMC Neurology*.

[22] Yang L., Jiang Q., Guan H., Bo H. (2019). Nursing care in anti-N-methyl-d-aspartate receptor encephalitis: a case series. *Medicine*.

[23] Dalmau J., Gleichman A. J., Hughes E. G. (2008). Anti-NMDA-receptor encephalitis: case series and analysis of the effects of antibodies. *The Lancet Neurology*.

[24] Graus F., Titulaer M. J., Balu R. (2016). A clinical approach to diagnosis of autoimmune encephalitis. *The Lancet Neurology*.

[25] Ogata M., Satou T., Miyazaki Y., Otsuka E., Saito N. ., ..., Shirao K. (2019). Correlations of cytokine levels in cerebrospinal fluid and peripheral blood with outcome of HHV‐6B encephalitis after hematopoietic stem cell transplantation. *Transplant Infectious Disease*.

[26] Imaz A., Cayuela N., Niubó J. (2014). Short communication: focal encephalitis related to viral escape and resistance emergence in cerebrospinal fluid in a patient on lopinavir/ritonavir monotherapy with plasma HIV-1 RNA suppression. *AIDS Research and Human Retroviruses*.

[27] Baumer T., Fry C., Luppe S., Gunawardena H., Sieradzan K. (2017). Human herpes virus-6 encephalitis causing severe anterograde amnesia associated with rituximab, azathioprine and prednisolone combination therapy for dermatomyositis. *Journal of Neurovirology*.

[28] Vidaña B., Johnson N., Fooks A. R., Sánchez‐Cordón P. J., Hicks D. J., Nuñez A. (2020). West Nile Virus spread and differential chemokine response in the central nervous system of mice: role in pathogenic mechanisms of encephalitis. *Transboundary and Emerging Diseases*.

[29] Sovinz P., Schwinger W., Lackner H. (2010). Severe epstein-barr virus encephalitis with hemophagocytic syndrome. *Pediatric Infectious Disease Journal*.

[30] Sisinni L., Gasior M., de Paz R. (2018). Unexpected high incidence of human herpesvirus-6 encephalitis after naive T cell-depleted graft of haploidentical stem cell transplantation in pediatric patients. *Biology of Blood and Marrow Transplantation*.

[31] Singh D., Kumar V., Yadav V., Kaur M. (2020). Deep neural network-based screening model for COVID-19-infected patients using chest X-ray images. *International Journal of Pattern Recognition and Artificial Intelligence*.

[32] Gianchandani N., Jaiswal A., Singh D., Kumar V., Kaur M. (2020). Rapid COVID-19 diagnosis using ensemble deep transfer learning models from chest radiographic images. *Journal of Ambient Intelligence and Humanized Computing*.

